# A new synthetic derivative of cryptotanshinone KYZ3 as STAT3 inhibitor for triple-negative breast cancer therapy

**DOI:** 10.1038/s41419-018-1139-z

**Published:** 2018-10-27

**Authors:** Wenda Zhang, Wenying Yu, Guiping Cai, Jiawen Zhu, Chao Zhang, Shanshan Li, Jianpeng Guo, Guoping Yin, Chen Chen, Lingyi Kong

**Affiliations:** State Key Laboratory of Natural Medicines, Department of Natural Medicinal Chemistry, China Pharmaceutical University, 24 Tong Jia Xiang, 210009 Nanjing, China

## Abstract

Silencing STAT3 is confirmed as a promising therapeutic strategy for triple-negative breast cancer (TNBC) therapy to address the issue of its poor prognosis. In this study, the natural product cryptotanshinone was firstly remodeled and modified as a more effective STAT3 inhibitor by structure-based strategy. The synthetic derivative **KYZ3** had 22–24-fold increase in antitumor activity than cryptotanshinone on two TNBC cell lines but had little effect on normal breast epithelial MCF-10A cells. Further investigation showed that **KYZ3** inhibited persistent STAT3 phosphorylation. It also prevented the STAT3 protein nuclear translocation to regulate the expressions of the target oncogenes including Bax and Bcl-2. Furthermore, KYZ3 inhibited TNBC cell metastasis by decreasing the levels of MMP-9 which were directly regulated by activated STAT3. A STAT3 plasmid transfecting assay suggested that **KYZ3** induced tumor cell apoptosis mainly by targeting STAT3. Finally, **KYZ3** suppressed the growth of tumors resulting from subcutaneous implantation of MDA-MB-231 cells in vivo. Taken together, **KYZ3** may be a promising cancer therapeutic agent for TNBC.

## Introduction

Triple-negative breast cancers (TNBCs) are more likely to metastasize and have poor prognosis without effective drugs^1,2^. Inhibiting aberrantly activated signal transducer and activator of transcription (STAT) 3 in TNBCs may be a promising strategy^3,4^. STAT3 is classified as an essential oncogene that regulates a master of the cellular events, including cancer cell proliferation, apoptosis and metastasis^5–8^.

The activation of STAT3 is phosphorylated at Tyr705 residue mediated by growth factor receptor tyrosine kinases and the cytoplasmic kinases^9–12^. Two phosphorylated STAT3 proteins form homo-dimeric-activated transcription factor complex via reciprocal binding of pTyr-SH2 domains^13–18^. Subsequently, the complexes translocate to the nucleus and induce the target gene expression^19–23^. The SH2 domain of STAT3 possesses two “hot spots”, a pY705 site and a nearby pY+X site^24–26^. The pY705 site is a good starting point for drug design, which mainly consists of polar residues such as Lys591, Arg609, and Glu612 responsible for binding to pTyr705 residues. While the pY+X site is associated to the selectivity of STAT3 inhibitors. Therefore, targeting pY705 site and pY+X site is an effective strategy for designing new STAT3 inhibitors^27–33^. Some of STAT3 inhibitors are on the clinical research, while there is still no STAT3 inhibitor antitumor drugs in the market^34,35^.

Natural products are the treasure for drug development, which have been providing novel skeletons and biological compounds to develop new drugs^36–38^. Nearly 60% drugs in the market are directly or indirectly derived from natural compounds^39^. Cryptotanshinone is a bioactive component in dried roots Salviamiltiorrhiza Bunge (Danshen) and the subject of extensive research about its antibacterial activity and anti-inflammation activity. While Shin Dae-Seop and coworkers reported that cryptotanshinone but not Tanshinone IIA is a STAT3 inhibitor for the potent anticancer agent by directly targeting SH2 domain in 2009 year^40,41^. However, its moderate potency limits it to use for cancer therapy. Therefore, structural modification of cryptotanshinone is imperative and valuable to develop more potent STAT3 inhibitors for anticancer agents.

In this study, according to the literatures and structure analysis of the binding model in silico, a new series of STAT3 inhibitors were designed by structure-based drug design strategy, and then synthesized and biologically evaluated with enhancing activity. The most potent derivative **KYZ3** was elucidated as a new STAT3 inhibitor with antitumor activity against TNBCs in vitro and in vivo.

## Results

### KYZ3 was considered as a STAT3 inhibitor and exhibited more sensitivity to cancer cells

According to the literature and structure analysis of the binding model in silico, the saturated D ring of cryptotanshinone was essential moiety for its p-STAT3 inhibition. The methyl group on D ring was exposed to the outside of the protein surface into the water environment, which could weaken the interaction with STAT3 protein. The A ring of cryptotanshinone increased the rigidity and just bound above the side pocket of the SH2 domain, which led to the poor interaction. Based on these, we modified the A and D rings of cryptotanshinone as shown in Fig. 1a, a new series of STAT3 inhibitors **KYZ1-15** were designed by structure-based drug design, and then synthesized (Fig. 1b).

**Fig. 1:** Compound **KYZ3** was designed as a STAT3 inhibitor. **a** The design strategy and synthetic routes of the cryptotanshinone derivatives. Compound **KYZ3** targeted the SH2 domain of STAT3 and exerted enhanced antiproliferation. **b** The synthetic route of **cryptotanshinone** derivatives. **c** The antiproliferative activity of **cryptotanshinone** and **KYZ3** on TNBC *P* < 0.001. **d** The binding mode of **cryptotanshinone** or **KYZ3** and STAT3 SH2 domain (PDB 1BG1) by AutoDock4.2. The carbon atoms of **cryptotanshinone** and **KYZ3** were colored magenta and the key residues were shown. Hydrogen bond distances were shown as green. **e** Cell viability percentage was measured by an MTT assay after treatment of STAT3 knockdown MDA-MB-231 cells with **KYZ3** for 48 h

Two STAT3 overactivated human TNBC cell lines (MDA-MB-231 and MDA-MB-468) were employed to test the activity of designed compounds with cryptotanshinone and BP-1-102 as the positive control by 3-(4,5-dimethylthiazolyl)−2, 5-diphenyltetrazoliumbro-mide (MTT) assays. The IC_50_ values were summarized in Supplementary Table S1. All the compounds exhibited more antiproliferative activity than cryptotanshinone and BP-1-102. Among them, the most potent compound **KYZ3** inhibited the growth of MDA-MB-231 and MDA-MB-468 cells with IC_50_ values of 0.68 μM and 0.86 μM, which had 22–24-fold improvement in antiproliferation activity than cryptotanshinone (Fig. 1c). What’s more, further study showed that **KYZ3** was less sensitive to normal human mammary epithelial cell line MCF-10A and normal human liver cell line L02 cells (Supplementary Table S2). The data showed that our inhibitor KYZ3 had little effect on the ability of MCF-10A cells up to 5.0 μM for 48 h. The IC_50_ of KYZ3 for MCF-10A cell line was 13.12 μM, which is 19-fold to the IC_50_ of KYZ3 for MDA-MB-231 cell line, 0.68 μM, indicating KYZ3 has certain selectivity over normal breast cell line and breast cancer cell line.

To further validate the important effect of STAT3 on **KYZ3**-induced cell growth inhibition, STAT3 siRNA was infected into MDA-MB-231 cells to block STAT3 and p-STAT3 (Tyr705), the expression of STAT3 and p-STAT3 (Tyr705) were both dramatically inhibited along with the decrease of cell viability. The cells that transferred siRNA were treated with **KYZ3** for another 48 h; cell viability was further decreased by **KYZ3** (Fig. 1e), because of its further ablation of p-STAT3. All these data indicated that a new derivative of cryptotanshinone, **KYZ3**, was capable of antitumor activity due to its downregulation of p-STAT3.

**KYZ3** featured much better activity than the parent molecule cryptotanshinone. To investigate the mechanism of the improved antitumor activity, firstly, the potential binding mode with the STAT3 protein was predicted by docking experiments. As Fig. 1d illustrates**, KYZ3** bound tightly to the STAT3 SH2 domain by forming an essential hydrogen bonding interaction with the Arg609 residue of STAT3 protein, which was similar to the binding modes of cryptotanshinone. In addition, the 2-methyl group of **KYZ3** fitted deeply into the pTyr705 pocket compared to the 3-methyl group of cryptotanshinone exposure to the water environment. Furthermore, the flexible side chain of **KYZ3** on B ring could tightly bind to the side pocket. Together, these data provided a rationale explaining the markedly increased activity of **KYZ3** as a STAT3 inhibitor.

### **KYZ3** inhibited the phosphorylation nuclear translocation of STAT3, and regulated the expression of STAT3 target oncogenes

The effect of **KYZ3** on STAT3 phosphorylation was investigated by the western blot analysis. MDA-MB-231 and MDA-MB-468 cells were incubated with **KYZ3** and the levels of p-STAT3 were then examined. **KYZ3** suppressed STAT3 phosphorylation at Tyr705 residue in a dose-dependent manner, but had no effects on the total STAT3 levels in both cell lines (Fig. 2a). Nuclear translocation of STAT3 plays a critical role in STAT3:STAT3/DNA complex formation and its target gene expression. The p-STAT3 protein was retained in both cytoplasm and nucleus in MDA-MB-231 cells treated without **KYZ3**. While treatment with **KYZ3** led to a significant decrease of the p-STAT3 level in nucleus and cytoplasm. The fluorescence intensity is weaker in the nucleus than cytoplasm in MDA-MB-468 cells; treatment with **KYZ3** led to a decrease of the p-STAT3 level both in the nucleus and cytoplasm, but mainly in the cytoplasm (Fig. 2b). To gain more insights into the mechanistic effects of **KYZ3** on the STAT3 pathway, its effect on the expression of STAT3-targeted genes was examined. **KYZ3** inhibited the expressions of Bcl-2, and increased the levels of Bax in a dose-dependent manner in both MDA-MB-231 and MDA-MB-468 cells (Fig. 2c, d).

**Fig. 2:** Compound **KYZ3** inhibited STAT3 activity. **a** Western blot analysis of p-STAT3 (Tyr705) and STAT3 in whole-cell lysates of equal total protein prepared from MDA-MB-231 and MDA-MB-468 cells treated with compound **KYZ3** for 24 h. **b** MDA-MB-231 and MDA-MB-468 cells were treated with **KYZ3**. For immunofluorescent assay, cells were fixed and stained with anti-phospho-STAT3 (p-STAT3) and DAPI before subjected to ImageXpress Micro Confocal analysis. Red or orange: p-STAT3; blue: nuclei; scale bar 20 μm. **c** Western blotting assay and **d** qPCR analysis of the levels of Bcl-2 and Bax in MDA-MB-231 and MDA-MB-468 cells treated with **KYZ3** for 24 h ***p < 0.001

### KYZ3 inhibited cancer cell migration and the expression of MMP-9 and MMP-2 proteins

Migration is directly or indirectly responsible for the majority of cancer deaths. Antimetastasis treatment is thus the key to cure cancer^42^. To investigate the inhibitory effect of **KYZ3** on tumor migration, a wound healing assay was performed. In the presence of **KYZ3** at 0.25 μM, the migration of MDA-MB-231 cells was effectively suppressed, and was almost inhibited at 0.5 μM **KYZ3** (Fig. 3a). Next, the trans-well invasion assay was further performed; a significant reduction in invasive ability at 0.25 μM of **KYZ3** and an almost cessation of cancer migration at 0.5 μM **KYZ3** were observed (Fig. 3b). Matrix metalloproteinase (MMP) enzyme MMP-9 and MMP-2 control the epithelial−mesenchymal transition, and their expression levels are directly regulated by the activated STAT3^3,4,43^. The effect of **KYZ3** on MMP-9 and MMP-2 expression levels was investigated. A dose-dependent decrease of MMP-9 and MMP-2 was induced by **KYZ3** (Fig. 3c, d). These data suggested that **KYZ3** inhibited cancer cell migration by decreasing the levels of MMP-9 and MMP-2.

**Fig. 3:** Compound **KYZ3** inhibited the cancer cell metastasis by decreasing MMP-9 levels. **a** The effect of **KYZ3** on tumor metastasis by wound healing assay (magnification, ×200). **b** The effect of **KYZ3** on tumor metastasis by trans-well migration assay (magnification, ×200). **c** Western blotting assay and **d** qPCR analysis of the levels of MMP-9 proteins in MDA-MB-231 cells ***p < 0.001, **p < 0.01. **e** Western blotting assay analyses the levels of p-STAT3 and the target gene expressions in MDA-MB-231 with STAT3 plasmid transfected by lentivirus

Previous experiments indicated that **KYZ3** inhibited the phosphorylation of STAT3. To investigate whether the effect of KYZ3 could be recovered partially with further overexpression of p-STAT3 in MDA-MB-231 cells, we transfected the MDA-MB-231 cells with further STAT3; thus the p-STAT3 level was also increased. As a result, **KYZ3** could inhibit p-STAT3 level but did not affect the total STAT3 level. The inhibition of the p-STAT3 level of the transfected cells was recovered a little bit upon treatment with 2 μM of **KYZ3** (Fig. 3e) **p < 0.01, ***p < 0.001.

### KYZ3 induced the ROS generation but did not inhibit the phosphorylation of the upstream kinases

The activation of STAT3 phosphorylated at Tyr705 residue may be mediated by the upstream kinases. The effect of **KYZ3** on p-Src and p-Erk protein levels was evaluated by the western blot analysis. Data showed that **KYZ3** had little effect on p-Src, and p-Erk expressions, indicating that the inhibition of **KYZ3** on p-STAT3 was not related with inhibiting p-Src and p-Erk (Fig. 4a).

**Fig. 4:** Compound **KYZ3** induced ROS generation without affecting the upstream kinases of STAT3. **a** Western blot analysis of p-Src and p-Erk levels in whole-cell lysates of equal total protein prepared from MDA-MB-231 and MDA-MB-468 cells treated with compound **KYZ3** for 24 h. MDA-MB-231 (**b**) and MDA-MB-468 (**c**) cells were incubated with **KYZ3** at different concentrations for 24 h, and then cells were collected and stained by DCFH-DA and subjected to flow cytometry. ***p < 0.001, **p < 0.01

The moderate level of reactive oxygen species (ROS) is sufficient for cancer cells to show active metabolism in response to oncogenic signal. In general, cancer cells take advantage of this moderate oxidative stress for proliferation, metastasis, and angiogenesis and so on. Nevertheless, high levels of ROS irreversibly damage DNA and lipids and ultimately cause cancer cell apoptosis^44^. The effect of **KYZ3** on the ROS levels in tumor cells was evaluated. The levels of ROS showed 1.2-, 1.3-, and 1.6-fold increases in MDA-MB-231 cells (Fig. 4b) and 1.1-, 1.4-, and 1.9-fold increases in MDA-MB-468 cells at 0.5, 1.0, and 2.0 μM of **KYZ3** (Fig. 4c), indicating that **KYZ3** induced ROS accumulation which may partially contribute to its selective inhibition on cancer cell proliferation and metastasis.

### KYZ3 induced breast cancer cell apoptosis but did not affect MCF-10A breast epithelial cells

The mechanism of cancer cell apoptosis induced by **KYZ3** was investigated. The effect of **KYZ3** on tumor cell apoptosis was analyzed by flow cytometry. Annexin V-APC/7-AAD staining was carried out and determined using flow cytometry. **KYZ3** dose-dependently induced the apoptosis of MDA-MB-231 and MDA-MB-468 cells. The induced apoptosis rates at 0, 1.0, 2.0, and 4.0 μM were 4.6, 33.9, 64.9, and 67.5% (Fig. 5a), and 2.9, 17.5, 26.2, and 47.1% (Fig. 5b), respectively. However, there was little apoptosis induced by **KYZ3** at 4.0 μM in MCF-10A cells (Fig. 5c), further indicating that **KYZ3** was a selective antitumor agent possibly through Bax/Bcl-2-related caspase-dependent apoptosis pathway by inhibiting STAT3 activity. Western blot analysis revealed that **KYZ3** increased the cleavage levels of PARP and Caspase3 proteins in MDA-MB-231 and MDA-MB-468 cells. Taken together, all these results further demonstrated that **KYZ3** induced cell apoptosis by targeting STAT3.

**Fig. 5:** Compound KYZ3 induced human carcinoma MDA-MB-231 and MDA-MB-468 apoptosis but not MCF-10A cells in vitro. MDA-MB-231 (**a**), MDA-MB-468 (**b**), and MCF-10A (**c**) cells were incubated with **KYZ3** at different concentrations for 24 h. Western blot analysis of cleaved-PARP and cleaved caspase3 levels in whole-cell lysates. Annexin V-APC/7-AAD staining was carried out and determined using flow cytometry. **p < 0.01, ***p < 0.001

### **KYZ3** exhibited antitumor activity in vivo

To evaluate the in vivo anticancer activity of **KYZ3**, BALB/c nude mice were inoculated subcutaneously with human breast cancer cells MDA-MB-231. Treatment with 15 mg/kg of **KYZ3** reduced the volumes of the implanted human breast tumor, while treatment with 30 mg/kg of **KYZ3** further inhibited the growth of the implanted tumors (Fig. 6a). Importantly, the weight of tumor tissues from mice treated with **KYZ3** was significantly reduced by 36.2 or 59.4%, and there was no significant body weight loss (Fig. 6b). Immunohistochemistry analysis of lysates from the tumor tissues treated with **KYZ3** showed a suppression of Ki67 compared with the control tumors (Fig. 6c) upon H&E staining. We stained Ki67 with H&E and quantified the Ki67 expression across a much larger field area. The results (Fig. 6c) showed that the inhibition of Ki67 expression in T1 was about 47% and in T2 was about 65%. We have investigated the levels of p-STAT3 in the control and treated tumors by immunohistochemistry. As Fig. 6d shows, KYZ3 inhibited the levels of p-STAT3 in vivo. These results showed that **KYZ3** had potent antitumor activity against the growth of implanted human breast tumors with little toxicity.

**Fig. 6:** Compound **KYZ3** inhibited the growth of human xenograft tumor in vivo. **a** The growing curves of mice’s tumor size. **b** The growing curves of mice’s body weight. **c** Immunohistochemical staining for Ki-67 in tumor tissues obtained from the control and **KYZ3**-treated mice. **d** **KYZ3** inhibited the levels of p-STAT3 in tumors ***p < 0.001, **p < 0.01, *p < 0.05

## Discussion

Triple-negative breast cancer is the leading cause of cancer-related morbidity and mortality in women. It is more likely to metastasize and have poor prognosis without special drugs^1^. Therefore, there is a paucity of effective treatments for managing patients with metastatic TNBCs^2^. Inhibiting aberrantly activated signal transducer and activator of transcription (STAT) 3 in TNBC may be a promising strategy for addressing this issue.

STAT3 is classified as an essential oncogene that regulates a master of the cellular events, including cancer cell proliferation, apoptosis, and metastasis^5–8^. The SH2 domain of STAT3 plays a critical role in the recruitment of STAT3 activation and the formation of STAT3 homodimers along with the formation of STAT3:STAT3/DNA complex^24,25^. Thus, designing STAT3 inhibitor targeting SH2 domain is an effective strategy to silence STAT3 activity^27–33^.

Natural products provide a varied and complex template structure for drug development. Cryptotanshinone is a bioactive component present in the dried roots of Salviamiltiorrhiza Bunge (Danshen), and was reported, in the year 2009, as a STAT3 inhibitor for the potent anticancer agent by directly targeting the SH2 domain^39,45^. However, its moderate potency limits its use for cancer therapy and its modification has not been reported till now.

This is the first study to report on the design, synthesis, and biological evaluation of cryptotanshinone analogs as new STAT3 inhibitors. According to the structure-based drug design strategy, a series of new STAT3 inhibitors were obtained. Especially, the derivative **KYZ3** exhibited 22–24-fold increase in antitumor activity against two typical TNBC cell lines with less sensitivity to MCF-10A cells and L02 cells. Docking studies discovered **KYZ3** targeted the STAT3 SH2 domain. Targeting this domain not only could inhibit STAT3 phosphorylation but also could suppress the STAT3:STAT3/DNA-binding complex forming which regulates downstream oncogene expression. Subsequently, the investigation of antitumor mechanism showed that **KYZ3** inhibited persistent and IL-6-induced STAT3 phosphorylation, STAT3 nuclear translocation and regulated the expression of STAT3 target genes such as Bax and Bcl-2. Bax/Bcl-2 are apoptosis genes; the increasing ratio of them induced by **KYZ3** activated the caspase-dependent apoptosis pathway of TNBCs. More importantly, **KYZ3** inhibited cancer cell metastasis by decreasing the expression of MMP-9, which were directly regulated by activating STAT3, suggesting that **KYZ3** may be a promising antimetastasis agent. Additionally, the ROS levels of cancer cells were increased by **KYZ3**, which further induced the tumor cell apoptosis and increased the antiproliferative selectivity against cancer cells. Furthermore, **KYZ3** in vivo induced significant antitumor responses, and exhibited no observed toxicity. In summary, **KYZ3** was confirmed as a new STAT3 inhibitor and exhibited marked antitumor activity, which is worthy of further investigation in order to develop effective STAT3 inhibitors for TNBC.

## Materials and methods

### Chemistry

The design and synthetic strategy for compounds **KYZ1-16** are shown in Fig. 1. Positive control cryptotanshinone and BP-1-102 was purchased from commercial suppliers. All of the cryptotanshinone derivatives were confirmed by ^1^H NMR, IR, HRMS (ESI) spectra, and ^13^C NMR spectrum, and are shown in Supplementary Materials and Methods.

### Docking

Computational docking program AutoDock4.2 was used to dock **KYZ3** to predict the binding mode. Briefly, compound **KYZ3** was docked using the Lamarckian Genetic Algorithm. The ligand and macromolecule were prepared using the Schrödinger software. Then, AutoGrid maps were prepared for all atom types. After 10 million energy evaluations were completed, the root-mean-square deviation threshold was set as 1.5 Å and all the resulting conformations of the ligands in the binding pocket of the macromolecule were clustered.

### Maintenance of cell lines culture and cell viability assays

All cell lines were purchased from Cell Bank of Shanghai Institute of Biochemistry and Cell Biology, Chinese Academy of Sciences (Shanghai, China). MtrDNA sequence analysis was done by the Cell Bank of Shanghai Institute of Biochemistry and Cell Biology, Chinese Academy of Sciences, Key GEN Bio TECH Co., Ltd., and Wuhan Gene Create Biological Engineering Co., Ltd. Human breast carcinoma cells MDA-MB-231 and MDA-MB-468, breast epithelial cells MCF-10A and human normal liver cells L02 were maintained in RPMI-1640 medium. All cells were supplemented with 12% fetal bovine serum containing 50 μg/mL penicillin and 50 μg/mL streptomycin. Cells were grown to 80% confluency in a tissue culture flask at 37 °C in a humidified atmosphere containing 5% CO_2_, and then were trypsinized and splitted.

Cells were seeded in 96-well plates at a density of 3000–6000 cells per well. The cells were incubated at 37 °C overnight. After medium removal, different concentrations of test compounds were added in triplicate to the plates in 200 μL fresh mediums; the plates were incubated at 37 °C for 72 h. Then 20 μL MTT was added to evaluate cell viability. The absorbance was read by an ELISA reader (SpectraMax Plus384, Molecular Devices, Sunnyvale, CA) at a test wavelength of 570 nm and a reference wavelength of 630 nm. Cell viability was calculated by the following formula:

$$\% \,{\mathrm{Cell}}\,{\mathrm{viability}} = \left( {{\mathrm{At}}/{\mathrm{As}}} \right) \times 100\%.$$

At and As denoted the absorbance of the test substances and solvent control, respectively.

### Western blot analysis

Cells were incubated with various concentrations of **KYZ3** for 24 h. Harvesting after trypsinisation, cells were treated with 1× RIPA lysis buffer (50 mM Tris-HCl, pH 7.4, 150 mM NaCl, 0.25% deoxycholic acid, 1% NP-40,1 mM EDTA and protease inhibitors) (Amresco, Solon, USA) to extract the total proteins. An aliquot of proteins from the total cell lysates (30−60 μg/lane) was separated by sodium dodecyl sulfate (10%) polyacrylamide gel electrophoresis (SDS-PAGE, BioRad Laboratories, Hercules, CA), wet-transferred to NC membrane (BioRad Laboratories, Hercules, CA) and blotted with primary antibodies specific for STAT3, p-STAT3, p-Src, P-Erk, Cleaved-PARP, PARP, Cleaved Caspase3, Caspase3, Bcl-2, Bax, MMP-9, and GAPDH. Bound immuno-complexes were detected using Chemi DOC™ XRS+ system (BioRad Laboratories, Hercules, CA).

### Immunofluorescence staining assays

Cells (1×10^4^/well) were cultured on 96-well glass culture plate (Corning, USA). After incubation with different concentrations of **KYZ3**, cells were fixed with 4% paraformaldehyde for 15 min, and permeabilized with 0.5% Triton X-100 for 15 min. Next, the cells were blocked with 5% BSA for 1 h and incubated with the primary antibody overnight at 4 °C. Alexa-conjugated secondary antibodies (Alexa Fluor 594 goat anti-rabbit IgG, Alexa Fluor 488 goat anti-rabbit IgG, Cell Signaling Technology, MA, USA) were applied and incubated at room temperature for 1 h. Cell nucleus was stained with 4, 6-diamino-2-phenyl indole (DAPI, Cell Signaling Technology, MA, USA) for 10 min. Finally, the cells images were analyzed by ImageXpress® Micro Confocal (Molecular Devices, USA).

### Quantitative real-time RT-PCR

Levels of mRNA expression were analyzed with the RT-PCR assay, with total RNA isolated from cells using an EASY spin Plus tissue/cell RNA extraction kit (Aidlab Biotechnologies Co. Ltd). RNA was quantified by measuring absorption at 260 nm and 1 μg of RNA was reverse transcribed to cDNA using the Transcriptor First Strand cDNA Synthesis Kit (Roche Diagnostics, Basel, Switzerland). Thermal cycling conditions included 95 °C initial denaturation for 5 min, followed by 40 cycles of denaturation (10 s at 95 °C), annealing (15 s at 60 °C) and extension (15 s at 72 °C with a single fluorescence measurement), a melt curve program (60–95 °C with a 0.11 °C/s heat increase and continuous fluorescence measurement) and a cooling step to 40 °C. The Δ cycle threshold method was used for the calculation of relative differences in mRNA abundance with a Light Cycler 480 (Roche Molecular Biochemicals, Mannheim, Germany). The data were normalized to the expression of GAPDH. The results were expressed as fold-changes. The RT-PCR primers that were used in this study are listed in the supporting information.

### Wound healing assays

Cells were seeded at 6×10^5^ cells per well into six-well plate and allowed to grow overnight. Wounds were made by scratching the cells with pipette tips (1–10 μL). Cells were treated with **KYZ3** and allowed to migrate into the scratched area for 24 h. The migration of cells was visualized at ×10 magnification using a Leica Microscope at time 0 h (immediately before the drug was added) and 24 h.

### Trans-well invasive assays

Cells were seeded at 3×10^4^ cells per well and allowed to grow overnight. The following day, the cells were serum-starved. Cells were treated with **KYZ3** and allowed to migrate into the scratched area for 24 h after being fixed in 4% paraformaldehyde for 10 min. Crystal violet solution (Sigma, St. Louis, MO, USA) was used to stain the colonies for 4 h. The migration of cells was visualized at ×10 magnification using a Leica Microscope.

### Apoptotic assay

Cells at a density of 2.5×10^5^ per well were cultured in regular growth medium in six-well plates for 24 h and treated in duplicate with different concentrations of **KYZ3** for 24 h. The cells were harvested, washed and stained with 5 μL Annexin V-APC and 5 μL 7-AAD at room temperature for 15 min. Cells were then analyzed by flow cytometry (488 nm excitation and 600 nm emission filters) using BD FACSCalibur flow cytometer (Becton & Dickinson Company, Franklin Lakes, NJ).

### Detection of ROS

Cells were seeded at a density of 3×10^5^ per well of six-well plates. The cells were treated with various concentrations of **KYZ3** for 24 h. The growth media was replaced with serum-free medium containing a final concentration of 10 μM DCFH-DA probe. After incubation for 20 min at 37 °C, cells were washed with serum-free medium twice, digested by trypsin and resuspended in the prewarmed PBS buffer. The samples were then subjected to a flow cytometry assay using BD FACSCalibur flow cytometer (Becton & Dickinson Company, Franklin Lakes, NJ).

### In vivo studies

Four-week-old, 20 g, female BALB/c nude mice (16–18 g) were injected with human breast tumor MDA-MB-231 (3×10^6^ cells in a volume of 0.2 mL) into the subcutaneous tissue of the mice. Three days after the tumor cell inoculation, the mice were randomly sorted into three groups with six mice per group. The tumor-bearing mice were either given an i.p. injection 15 mg/kg or 30 mg/kg of compound **KYZ3**. The treatment was initiated when the tumor burden of mice reached around 80 mm^3^. The tumor size was measured three times a week and calculated by the formula: length × width^2^/2, and the body weight was measured and recorded. On the 22nd day, all mice were killed, and the tumor was segregated, and weighed. The levels of p-STAT3 in tumor tissues were analyzed by the western blot assay.

The experimental mice were cared for and handled strictly according to the recommendations of the Animal Ethics Committee of China Pharmaceutical University, and the National Institutes of Health (NIH) standard guidelines for the Care and Use of Laboratory Animals. All experimental protocols were approved by the Animal Ethics Committee of China Pharmaceutical University.

### Statistical analysis

Statistical analysis was performed with ANOVA by using Graph Pad Prism version 5.0 (Graph Pad Software, San Diego, CA, USA). The results were given as the mean ± SD. *p* < 0.05 was considered significant.

## Electronic supplementary material

A new synthetic derivative of cryptotanshinone KYZ3 as STAT3 inhibitor for triple negative breast cancer therapy

Supplementary Table S1

Supplementary Table S2
